# Algorithm of Pulmonary Vascular Segment and Centerline Extraction

**DOI:** 10.1155/2021/3859386

**Published:** 2021-08-25

**Authors:** Shi Qiu, Jie Lian, Yan Ding, Tao Zhou, Ting Liang

**Affiliations:** ^1^Key Laboratory of Spectral Imaging Technology CAS, Xi'an Institute of Optics and Precision Mechanics, Chinese Academy of Sciences, Xi'an 710119, China; ^2^Department of Pathology, The First Affiliated Hospital of Xi'an Jiaotong University, Xi'an 710061, China; ^3^Changshu Institute of Technology, Suzhou 215500, China; ^4^School of Computer Science and Engineering, North Minzu University, 750021 Yinchuan, China; ^5^Department of Radiology, The First Affiliated Hospital of Xi'an Jiaotong University, Xi'an 710061, China; ^6^Science and Technology Department, The First Affiliated Hospital of Xi'an Jiaotong University, Xi'an 710061, China

## Abstract

Because pulmonary vascular lesions are harmful to the human body and difficult to detect, computer-assisted diagnosis of pulmonary blood vessels has become the focus and difficulty of the current research. An algorithm of pulmonary vascular segment and centerline extraction which is consistent with the physician's diagnosis process is proposed for the first time. We construct the projection of maximum density, restore the vascular space information, and correct random walk algorithm to satisfy automatic and accurate segmentation of blood vessels. Construct a local 3D model to restrain Hessian matrix when extracting centerline. In order to assist the physician to make a correct diagnosis and verify the effectiveness of the algorithm, we proposed a visual expansion model. According to the 420 high-resolution CT data of lung blood vessels labeled by physicians, the accuracy of segmentation algorithm AOM reached 93%, and the processing speed was 0.05 s/frame, which achieved the clinical application standards.

## 1. Introduction

In recent years, the air is in poor quality, which seriously affects people's life and health, resulting in an increasing incidence of lung cancer. Because the early symptoms of lung cancer are relatively minor, it is not easy to be discovered, and 80% of lung cancer patients are already in the middle and late clinical stage when they are confirmed, missing the best period of radical operation. If the lung cancer can be detected earlier and get differential diagnosis by category, it can receive standard treatment before the lesion spread, the patient's five-year survival rate can reach more than 60% [1, 2]. If the lung CT data which intuitively reflect the lung condition can be accurately analyzed, lung disease can also be prevented and diagnosed, and more human life can be saved. Pulmonary vascular lesions are one of the early signs of lung cancer, so accurate division and observation of pulmonary vascular areas are very important for diagnosis and treatment [3].

Due to the small morphological structure of pulmonary blood vessels and complex distribution environment, the process of imaging is easily affected by noise and surrounding tissues. This has brought great difficulty to the complete extraction of lung blood vessels, which is also the focus of the current research. According to the characteristics of the vascular section obeying Gaussian distribution, Foncubierta-Rodríguez et al. [4] constructed an enhancement model of vascular segmentation to determine the direction of vascular growth and extract blood vessels. According to the vascular anatomy, Orkisz et al. [5] calculated the global threshold to divide the lung image, and then, the blood vessels are extracted by discriminating the connectivity. Based on the two-dimensional CT image, Ibrahim et al. [6] selected the initial point manually, calculated the blood vessel position step by step, and then segmented the blood vessel. Lai et al. [7] enhanced the vascular response by filtering the image from a 3D angle. Gong et al. [8] extracted the blood vessels by constructing the self-adaptive threshold according to the difference between the gray level of the blood vessel and the surrounding area. Charbonnier et al. [9] constructed a matching model in accordance with blood vessels extending throughout the lungs to segment the blood vessels. Based on the local feature model, Gupta et al. [10] predicted the blood vessel direction. According to the samples of axial position, coronal position, and sagittal position, Phellan et al. [11] constructed a CNN model to segment the vascular area. Lidayová et al. [12] established the model of normal blood vessel and abnormal blood vessel to realize the segmentation of blood vessel. Jawaid et al. [13] improved level set to extract the vascular boundary information. Xiao et al. [14] used the grayscale and shape characteristics to constrain and segment blood vessels. Flórez and Orkisz [15] established the cylindrical model to simulate the distribution of blood vessels. Hu et al. [16] improved the crossaccess law function to extract blood vessels.

Because it is difficult for doctors to observe small changes of blood vessels through the naked eye to make accurate diagnosis, computer-assisted diagnosis is required. Based on the above extraction of the vascular centerline, the mainstream diagnostic method is as follows: adjust the window width and window position [17] when blood vessels are observed, the 3D model [18] shows the overall external morphology of blood vessels, a virtual endoscope [19] shows the inside of the blood vessels. The above algorithms cannot give the internal and external characteristics of blood vessels at the same time, which limited the ability of helping physician to diagnose.

The main problems of vascular division, centerline extraction, and auxiliary diagnosis can be summarized as follows: (1) the 3D model of extracting vascular segment is complex, and it needs a large amount calculation, so it cannot be calculated and displayed in real time; (2) it is difficult to divide the vascular area accurately just by gray scale; and (3) there is no accurate and intuitive way to show the internal and external conditions of blood vessels.

For those reasons, we study the process of doctors' diagnosis of vascular lesions and construct a diagnostic model for doctors' vision diagnosis according to the theory of medicine, anatomy, and image graphics: (1) establish a maximum density projection model based on vascular anatomy and imaging principles and significantly reduce the amount of data while retaining the area where the blood vessels are located; (2) adaptive random walk algorithm is constructed by combining gray level with local information; and (3) construct the mechanism of vascular centerline extraction and vascular expansion and display and diagnose vascular from multiangle.

## 2. Details of Algorithm

When physicians detect pulmonary vascular lesions, removing the interference of the examination bed, muscles, and soft tissues is the first task. They focus on the lung parenchyma and then determine the starting and ending points of the blood vessels to be observed based on the local images of limited frames, achieving the extraction of blood vessels. Finally, they extract the vascular centerline and give diagnosis based on the anatomical knowledge.

The computer simulates how doctors diagnose lesions as follows: the lung image sequence was firstly pretreated to remove noise and check a bed, and the image was simplified by extracting the lung parenchyma area. Then, it determined the starting and ending points of blood vessels to be observed using global and local models to constrain them and took the characteristics of anatomy and image graphics into consideration to realize the extraction of blood vessels' central line.  Figure 1 shows the flow of pulmonary vascular CAD segmentation.

### 2.1. Pretreatment

CT images can intuitively show the morphological structure of human tissues (blood vessels, musculoskeletal, etc.). According to the physician's diagnosis process, the blood vessels that physician concerned only exist in the lung parenchyma. The ends of the blood vessels are tiny; they are only displayed as a limited number of pixels in the image and are vulnerable to noise. Therefore, the image needs to be preprocessed.

#### 2.1.1. Noise Reduction

CT image always includes pepper and salt noise [20] which presented as a bright discrete pixel; it interferes with the extraction of pulmonary blood vessels' tip and needs to be removed. According to the characteristics that noises are distributed as discrete points, a two-dimensional median filtering algorithm can be used to remove them. The formula is as follows:

(1) $$\begin{array}{c} g\left(x,y\right)=\text{med }\left\{f\left(x-k,y-m\right),\left(k,m\in W\right)\right\}, \end{array}$$

where *f*(*x*, *y*) and *g*(*x*, *y*) are the gray values of the pixels with coordinates (*x*, *y*) in the original image and the processed image, respectively; *W* is a two-dimensional filter template; and med is a median filter function.

#### 2.1.2. Lung Parenchyma Extraction

The area of blood vessels that doctors care about is inside the lung parenchyma. Whether the extraction of the blood vessels is good or bad directly affects the subsequent diagnosis. Therefore, the computer needs to focus on the area where the pulmonary nodules are located. By analyzing the statistical distribution of lung image pixels, Qiu et al. [21] constructed an optimized Gaussian dual-mixing model to calculate the global segmentation threshold quickly, and the complete lung parenchyma region can be extracted. In order to meet the clinical application standards of accuracy and processing speed, the algorithm in literature [21] is applied to extract the lung parenchyma region and confirm the left and right lung regions.

#### 2.1.3. Set the Starting and Ending Points of Blood Vessels

When the doctor identifies the focal point, he will determine the observed vascular area through clinical needs. When the computer simulates this process, according to the morphological structure of blood vessels, it sets the blood vessel's starting point *P*_*b*_ and the end point *P*_*e*_ whose corresponding coordinates are (*x*_*b*_, *y*_*b*_, *z*_*b*_) and (*x*_*e*_, *y*_*e*_, *z*_*e*_) on the computer image through human-computer interaction, and *z*_*b*_ ≤ *z*_*e*_.

### 2.2. Rough Extraction by a Local 3D Model

The physician only cares about the blood vessel between point *P*_*b*_ and point *P*_*e*_, so the blood vessel area needs to be extracted.

Since blood vessels are of connectivity, as shown in Figure 2, only handle [*z*_*b*_, *z*_*b*_ + 1, ⋯*z*_*e*_] is not rigorous, where *m* is the point on the blood vessel.

Anatomically, blood vessels are spatially continuous. From the perspective of image imaging, blood vessels appear as bright and isolated circular areas in two-dimensional CT images.

In order to restore the anatomical characteristics of blood vessels, we introduce the maximum density projection which is integrated with the local 3D information to greatly reduce the amount of data while ensuring the information of blood vessels.

The maximum intensity projection is a method for 3D data that projects in the visualization plane the voxels with maximum intensity that fall in the way of parallel rays traced from the viewpoint to the plane of projection. The equation is as follows:

(2) $$\begin{array}{c} {MIP}_{n}\left(x,y\right)=\max\left(I_{k+1}\left(x,y\right)\cdots I_{k+{\text{SN}}_{r}}\left(x,y\right)\right),\\ 1\leq x\leq H,\\ 1\leq y\leq W,\\ k=\left(n-1\right)\times {\text{SN}}_{r},\\ n=1,2\cdots \frac{\text{Nm}}{{\text{SN}}_{r}}, \end{array}$$

where **MIP***n*(*x*, *y*) is the grayscale value at the midpoint (*x*, *y*) of the *n*th frame of the MIP image; *H* and *W* are the horizontal and vertical resolutions, respectively; SN_*r*_ is the number of projected layers; and Nm is the sum of original CT layers. *I*_*k*_(*x*, *y*) is the grayscale value at the point (*x*, *y*) in the *k*th layer of the original CT sequence images.  Figure 3 is a schematic diagram of the MIP projection of the two-dimensional CT data.

The blood vessels in the MIP image are locally highlighted and continuous areas, as shown in Figure 4(a). Subsequent extraction of vascular areas is needed to constrain the vascular centerline method and reduce the amount of data. In the MIP image, *P*_*b*_ and *P*_*e*_ are chosen as seed points, The area of the blood vessel is obtained by using *C*-means clustering [22, 23], and then, the image of the suspected area *I*_*i*_ as Figure 4(b) is obtained through the 8 connected areas. Follow-up study is based on *I*_*i*_.

### 2.3. Segment by Automatic Random Walk Algorithm

Random walk (RW) algorithm [24] regarded the two-dimensional image as a connected undirected weighted graph containing fixed vertices and edges. The unlabeled pixels begin to walk along the edge from the vertices. According to the maximum probability of each pixel arriving at each labeled pixel, the class of each vertex is judged.

The main steps are (1) manually mark the seed point; (2) establish a random walk model *G* = (*V*, *E*), where *V* is the set of vertices of the image and *E* is the set of undirected edges at any two vertices of the image; (3) calculate weights; and (4) compute the distribution of probability and get the segmentation.

In recent years, Dong et.al [25] introduced subMarkov to realize image segmentation. Zheng et al. [26] constrain RW according to target characteristics. Bui et al. [27] established a 3D model to realize the heart division. All of the above methods get good results. As blood vessels run through multiple layers of images, it is inefficient to manually mark seed points on each layer of images. In a 2D image, blood vessels are shown as limited sections of pixels, and the number of pixels is small, so the accuracy of seed selection will directly affect the segmentation effect. For this reason, we study the selection of seed and weight calculation and then propose an algorithm.

#### 2.3.1. Adaptive 3D Seed Selection

The traditional RW algorithm segments the image semiautomatically. The user needs to manually mark the target seed and background seed on the 2D image, and then, the probability of each vertex to these two kinds of seed is used to judge which one they belong to, thus dividing the image into the target area and the background area.

The blood vessel exists on the CT image as a circular or cylindrical section. When using the traditional RW algorithm, the physician needs to spend a lot of time on accurately marking the seed on each 2D image. Besides, the number of blood vessel pixels is limited; the physician may mark the wrong seed because of a slight deviation, which cannot guarantee the completeness of the segmentation.

According to the characteristics of angiology, anatomy, and CT imaging, we optimize the process of selecting seeds as Figure 5. From the medical point of view, the components contained in the blood vessels are uniform, so the pixel values are similar in CT image. Anatomically, it is a continuous region in a 3D space. From the aspect of imaging, blood vessels are locally bright area.

The approximate area of the blood vessel in the 3D space is marked as *I*_*i*_, with the point *P*_*i*_ (*P*_0_ = *P*_*b*_) as the target seed and the nonvascular region in *I*_*i*_ as the background seed, and the divided blood vessels of the current layer was recorded as *C*_*i*_. According to the continuity of vascular, *C*_*i*_∩*C*_*i*+1_ ≠ ∅, according to the uniformity of blood composition, the pixel value of the blood vessel should change a little; then, the coordinate of the central point of *C*_*i*_∩*C*_*i*+1_ is assigned as *P*_*i*+1_.

#### 2.3.2. Calculate Weights

The weights determine that the probability of each vertex belongs to different classes. The traditional RW algorithm only considers the grayscale information between pixels and does not consider the geometric information between pixels. For more accurate segmentation, the improved weight function is

(3) $$\begin{array}{c} w_{i,j}=\exp\left(-\alpha \left|g\left(v_{i}\right)-g\left(v_{j}\right)\right|+\left(1‐\alpha \right)\left|h\left(v_{i}\right)-h\left(v_{j}\right)\right|\right),\\ L_{i,j}=\left\{\begin{array}{cc} d_{i}, & i=j,\\ -w_{i,j}, & v_{i}\text{ is adjacent to }v_{j},\\ 0, & \text{others}, \end{array}\right. \end{array}$$

where *g*(.) represents the grayscale, *h*(.) represents the coordinate value, *α* is the weight of grayscale, (1 − *α*) is the weight of distance, and *L*_*i*,*j*_ is the matrix of distance. RW algorithm is rebuilt to realize the automatic segmentation of blood vessels. The selected seeds are few, the calculation area is small, and the speed is fast. It reduces the workload of doctors and improves the diagnostic efficiency.

### 2.4. Centerline Extraction and Expansion

After the doctor confirms the vascular area, he reconstructed the 3D characteristics of the blood vessels and set up the center point to observe the pathological conditions of the blood vessels.

Because the spacing of CT data layers and the image resolution are not uniform, in order to restore the true situation of the lungs, the computer needs to interpolate the data to develop the isotropic data; that is, the lung data observed from any direction are uniform. According to MIP image processing, it can be seen that the space of blood vessels is limited, so it needs to be interpolated. The gray scale of the point *P*_*i*_ is used as the seed to cluster on the corresponding layer of the original image sequence to obtain the blood vessel area, whose center and the inscribed circle's radius *R* are calculated. Then, the point *P*_*i*_ in the image is seen as the center of the ball with a radius of 2*R*; the data sequence is interpolated vertically according to the resolution of the axis to form isotropic data.

Calculate the three eigenvalues *λ*_1_, *λ*_2_, and *λ*_3_ and the eigenvectors *ν*_1_, *ν*_2_, and *ν*_3_, which represent the trend of movement in different directions, as shown in Figure 6. Take *ν*_1_ as the blood vessel direction and 2*R* as the search radius; make some adjustment *R* to find the position of next blood vessel to obtain a complete blood vessel area.

In the process of the calculation, the following four situations occur, as shown in Figure 7, in which the red strip is a blood vessel and the balls show the adjustment process of centerline.

**Case 1 .**

Start off from *P*_*b*_; calculate *ν*_1_. In the direction of *ν*_1_, jump with the step 2*R*_0_. Calculate the coordinates of the center of ball's gravity *P*_1_ and radius *R*_1_ and save it.

**Case 2 .**

Start off from *P*_1_; calculate *ν*_1_. In the direction of *ν*_1_, jump to *P*_1_′ with the step 2*R*_1_. Constantly adjust the center of gravity and radius until they do not change; save the center of gravity *P*_2_ and radius *R*_2_.

**Case 3 .**

Start off from *P*_2_; calculate *ν*_1_. In the direction of *ν*_1_, jump to *P*_2_′ with the step 2*R*_2_, and the circle centered on *P*_2_′ with the radius *R*_2_ which is not in the MIP image, indicating that the step length is too large, which needs to be adjusted. When the cross section of circles reaches 10%, the step length is set to *R*_2_′. The coordinates at this point are *P*_2_^″^. Adjust the center of gravity and radius continuously until they do not change; save the center of gravity *P*_3_ and radius *R*_3_.

**Case 4 .**

Start off from *P*_3_; calculate *ν*_1_. In the direction of *ν*_1_, jump to *P*_3_′ with the step 2*R*_3_. If *P*_*e*_ is exceeded, take *P*_*e*_ as the center of the circle and adjust the length of the step, and the center of gravity of the ball is calculated and saved.

When the physician determines the vascular centerline, he needs to observe the internal and external conditions of the blood vessel; this process is simulated by the computer as follows: first, the blood vessels are straightened according to the centerline, and then, according to the anatomical principles, the blood vessels are expanded according to different profiles (0°, 45°, 90°, and 135°). The internal and external conditions of different profiles are observed to give a comprehensive judgment. Its schematic diagram is shown in Figure 8.

## 3. Experiments and Result Analysis

The experiment used 50 sets of CT data with different resolutions and thickness collected in 2020; 420 blood vessel areas were extracted. The programs were compiled in VS2015 with the WIN7 operating system.

### 3.1. Verify the Effect of MIP Algorithm

The same group of CT sequences was reconstructed as the layer thickness is 3 mm, 9 mm, and the entire sequence, respectively, by the MIP algorithm and compared with the original sequence. The effect is shown in Figure 9. The MIP algorithm can restore the strip shape of vascular and reduce the risk of wrong detection. With the increase of layer thickness, it can display the distribution of peripheral blood vessels more clearly and ensure that the follow-up extraction of vascular centerlines is more complete.

### 3.2. The Effect of Vascular Segmentation

To verify the effect of blood vessel extraction, three experts who have been engaged in medical imaging for many years were asked to mark blood vessels to verify the effect of the algorithm from the quantitative and qualitative levels.

The quantitative aspects are as follows: take area overlap measure (AOM) [28] as an evaluation indicator of the segmentation effect; it is defined as

(4) $$\begin{array}{c} \text{AOM}\left(A,B\right)=\frac{S\left(A\cap B\right)}{S\left(A\cup B\right)}\times 100\%, \end{array}$$

where AOM is the area overlap measure, *A* is the image marked by the doctor, *B* is the image segmented by computer, and *S*(·) represents the number of pixels in the corresponding area. The larger the AOM value is, the better effect the segmentation gets. The results are shown in Table 1.

The qualitative aspects are as follows: using medical diagnostic marks: “accurate” means that the vascular division is complete and almost identical with the area marked by experts; “general” indicates that there is a some deviation between the results of the two, but it does not affect the diagnosis; and “poor” indicates that there is a large deviation between the results of the two, which affects the diagnosis. The results are shown in Table 2.

This paper uses the Contrast-Enhanced (CE) algorithm [4] from both qualitative and quantitative aspects to construct a vascular enhancement model and achieve vascular segmentation. 3D algorithm [7] established a 3D model from the inside of the blood vessels. Multidirectional (MD) algorithm [11] observed the blood vessels from the axial, coronal, and sagittal direction, determined the direction of blood vessels, and then segmented them. Level set (LS) algorithm [13] transformed the segmentation problem into the problem of internal and external forces' balance. RW [24] selected the seed points manually on each layer of images to achieve vascular segmentation, not considering the time spent. Our algorithm takes full account of vascular anatomy and imaging principles, proposes an automatic selection algorithm for seed points, and optimizes the weight function; although a little more time was spent than CE [4] algorithm, the segmentation effect AOM reached 93%, and the effect that achieves the “general” was the best, thus confirming the effectiveness of the proposed algorithm.

To demonstrate the effect of our algorithm, we extract the whole pulmonary blood vessels. It is very difficult. The algorithm proposed in this paper can extract most of the blood vessels, but there are still some incomplete blood vessels extracted. As shown in Figure 10(b), the blood vessels are not completely extracted in the area where they enter the lungs. The main reason is that the left and right lungs of this sequence are relatively close. During the CT imaging process, the left and right lungs are not effectively divided. Further research is needed on this issue.

### 3.3. The Extraction of Vascular Centerline

In order to verify the effect of the extraction of vascular centerline and show the observation effect of the current major assisted diagnosis method, our algorithm, 3D display, and virtual insight are compared. The 3D display is shown in Figure 11(a); only the external condition of the blood vessel can be observed; the virtual insight is shown in Figure 11(b); only the internal condition of the blood vessel can be observed; and our algorithm is shown in Figure 11(c), which shows the inside and outside of the blood vessel at the same time and intuitively shows the effect of extraction of vascular centerline.

In order to intuitively demonstrate the effect of vascular expansion, we chose unbranched blood vessels, branching blood vessels, and blocked blood vessels, which were displayed at 0°, 45°, 90°, and 135°. Unbranched blood vessels, as shown in Figure 12, are spread in different directions; the centerline is in the center of the blood vessel. For branching blood vessels, as shown in Figure 13, the longest blood vessel (red) and the shortest blood vessel (blue) are selected for straightening. It can be seen that this algorithm is not affected by the blood vessels next to the branch when extracting the central line. The central line can be extracted accurately. Figures 12 and 13 show the effects of normal vascular centerline's extraction and spread, and the interior of blood vessel is relatively smooth.  Figure 14 shows the spreading effect of blocked blood vessel. It can be seen that the algorithm can accurately extract the centerline, and a lot of blocked spots can be observed inside the blood vessels. From the above demonstration, the algorithm presented in this paper can accurately extract the vascular centerline and directly display the internal and external conditions of blood vessels, so it can assist the physician to make an accurate diagnosis.

## 4. Conclusion

Computer-aided detection of pulmonary blood vessels has become a hot topic and difficulty in research. In this paper, the segmentation algorithm of pulmonary vascular CT image is proposed, which combines local 3D information and enhances vascular area. Optimize the random walk algorithm to meet the requirements of separating blood vessel accurately. We applied the knowledge of pathology, anatomy, and image graphics to the vascular centerline extraction and proposed the method of spreading blood vessels which can show the internal and external characteristics of blood vessels more clearly, thus assisting physicians in making accurate diagnoses. It is of great value on clinical application and lays a good foundation for the follow-up detection of vascular lesions. However, the vascular division is incomplete when the left and right lungs are near, and further research is needed.

## Figures and Tables

**Figure 1:** Algorithm flow chart.

**Figure 2:** Vascular route diagram.

**Figure 3:** MIP schematic.

**Figure 4:** MIP image processing: (a) MIP image; (b) *I*_*i*_.

**Figure 5:** Seed selection process.

**Figure 6:** Directional diagram of feature vector.

**Figure 7:** Vascular division: (a) Case 1, (b) Case 2, (c) Case 3, and (d) Case 4.

**Figure 8:** Vascular centerline expansion diagram.

**Figure 9:** The effect of reconstructing MIP diagram: (a) original image, (b) 3 mm, (c) 9 mm, and (d) entire sequence.

**Figure 10:** Full sequence segmentation results. (a) Segmentation results are “accurate.” (b) Segmentation results are “poor.”

**Figure 11:** Performance of the algorithm.

**Figure 12:** Effect of spreading unbranched blood vessel.

**Figure 13:** Effects of spreading branching blood vessels.

**Figure 14:** Effect of spreading blocked blood vessels.

**Table 1:** Quantitative evaluation of vascular segmentation.

Algorithm	AOM%	Average time (s/frame)
CE	73	0.03
3D	79	0.40
MD	83	0.07
LS	86	0.10
RW	85	—
Ours	93	0.05

**Table 2:** Qualitative evaluation of vascular segmentation.

Algorithm	Accurate	General	Poor
CE	223	139	58
3D	258	125	37
MD	265	136	19
LS	280	119	21
RW	225	159	36
Ours	312	93	15

## Data Availability

Data is available at International Early Lung Cancer Action Project (DB/OL) (http://www.via.cornell.edu/lungdb.html).
